# Effect of Cinepazide Maleate on Serum Inflammatory Factors of ICU Patients with Severe Cerebral Hemorrhage after Surgery

**DOI:** 10.1155/2021/6562140

**Published:** 2021-10-28

**Authors:** Jing Zhang, Xia Zhang, Yun Shang, Li Zhang

**Affiliations:** ^1^Department of Internal Medicine-Neurology, Linyi Central Hospital, Linyi 276400, Shandong Province, China; ^2^Endoscopy Room, The Fourth People's Hospital of Jinan, Jinan 250031, Shandong Province, China; ^3^Department of Equipment, Tai'an Maternal and Child Health Hospital, Tai'an 271000, Shandong Province, China; ^4^Department of Nursing, The First Affiliated Hospital of Shandong First Medical University, Shandong Province Qianfoshan Hospital, Jinan 250014, Shandong Province, China

## Abstract

**Objective:**

To explore the effect of cinepazide maleate on serum inflammatory factors of intensive care unit (ICU) patients with severe cerebral hemorrhage after surgery.

**Methods:**

116 ICU patients with severe cerebral hemorrhage treated in Taian Maternal and Child Health Hospital from June 2018 to June 2020 were selected as the research objects and randomly divided into the control group and experimental group, with 58 patients in each group. The control group was given routine treatment, while the experimental group was additionally given an intravenous drip of cinepazide maleate to compare the clinical efficacy and serum inflammatory factors between the two groups.

**Results:**

The total effective rate in the experimental group was higher than that in the control group (*P* < 0.05). After treatment, the Glasgow Coma Scale (GCS), National Institutes of Health Stroke Scale (NIHSS), and Fugl-Meyer scores in both groups were better than those before treatment, and the scores in the experimental group were better than those in the control group (*P* < 0.05). The oxidative stress indexes such as total antioxidant capacity (T-Aoc), superoxide dismutase (SOD), and glutathione peroxidase (GSH-PX) in the experimental group were higher than those in the control group, while malondialdehyde (MDA) in the experimental group was lower than that in the control group (*P* < 0.05). The high-sensitivity C-reactive protein (hsCRP), interleukin-6 (IL-6), interleukin-8 (IL-8), and tumor necrosis factor-*α* (TNF-*α*) levels in the experimental group were lower than those in the control group (*P* < 0.05). Compared with the control group, the cerebrovascular function in the experimental group was significantly improved (*P* < 0.05), with statistically significant differences.

**Conclusion:**

Cinepazide maleate can effectively reduce the serum inflammatory factor levels of ICU patients with severe cerebral hemorrhage after surgery, alleviate the oxidative stress response in the body, and improve the cerebrovascular function and cerebral nerve function, which is worthy of clinical promotion.

## 1. Introduction

Cerebral hemorrhage (also known as spontaneous intracerebral hemorrhage) refers to nontraumatic primary intraparenchymal hemorrhage, accounting for about 20%–30% of acute cerebrovascular diseases [1–4]. According to clinical statistics, about 80% of patients have cerebral hemorrhage in the cerebral hemisphere, with the remaining 20% in the cerebellum and brainstem. Cerebral hemorrhage is a type of acute cerebrovascular disease with the highest mortality rate, mostly in elderly patients over 50 years old or in patients with a history of hypertension. In clinical treatment, most patients receive medical treatment. In the acute phase, bleeding control and reducing intracranial pressure are the main measures, and supportive medical care is necessary after cerebral hemorrhage is stopped [5–8]. Cinepazide maleate is a calcium channel blocker to inhibit Ca^2+^ influx, relax the vascular smooth muscle, and dilate coronary arteries. In clinical studies, animal experiments have confirmed that this substance has a certain inhibitory effect on the inflammatory response in the process of focal cerebral ischemia-reperfusion injury in rats, protecting the brain [9–12]. In recent years, the medical research about cinepazide maleate mostly focuses on its effect on hypertensive cerebral hemorrhage (HICH) and lacks studies on severe cerebral hemorrhage. To further clarify the clinical effect of cinepazide maleate on patients with severe cerebral hemorrhage, this paper explored the effect of cinepazide maleate on serum inflammatory factor levels of ICU patients with severe cerebral hemorrhage after surgery, summarized as below.

## 2. Materials and Methods

### 2.1. General Information

116 ICU patients with severe cerebral hemorrhage treated in Taian Maternal and Child Health Hospital from June 2018 to June 2020 were selected as the research objects and randomly divided into the control group and experimental group, with 58 patients in each group.

### 2.2. Inclusion Criteria

(1) The patient met the diagnostic criteria in the *Guidelines for the Management of Spontaneous Intracerebral Hemorrhage* [13] and was confirmed by head CT and MRI examinations. (2) It was the first time that the patients had the disease, and if not the first time, there should be no residual neurological impairment after the first onset. (3) The onset time was no more than 24 hours. (4) The patients had clear consciousness and were able to cooperate with examination and treatment. (5) This study was approved by the ethics committee of Taian Maternal and Child Health Hospital, and the patients and their families accepted the treatment plan and signed informed consent.

### 2.3. Exclusion Criteria

(1) The patients had severe heart, lung, kidney, and liver dysfunction and were complicated with autoimmune diseases, hematological diseases, connective tissue diseases, or malignant tumors. (2) The patients had severe hypertension that could not be effectively controlled. (3) The patients had taken drugs affecting inflammatory response in the past one month. (4) The patients were allergic to drugs used in the study. (5) The patients refused to cooperate with researchers.

### 2.4. Methods

The control group received routine treatment measures immediately after admission, specifically as follows. (1) Dehydration: the patients with cerebral edema received 250 ml of 20% mannitol injection (specification: 250 ml/bottle; manufacturer: Shandong Wego Pharmaceutical Co., Ltd.; SFDA approval no. H20053865) by intravenous drip, 1-2 times a day. The dosage and treatment courses could be adjusted according to the severity of cerebral edema [14]. (2) Anticoagulation: 5000 IU of low-molecular-weight heparin calcium (1.0 ml: 5000 Axa unit; manufacturer: Shenzhen Scriprogen Biopharmaceutical Co., Ltd.; SFDA approval no. H20060190) was injected subcutaneously into the abdominal wall around the umbilicus every 12 hours. 80 mg of ozagrel sodium (specification: 40 mg; manufacturer: Youcare Pharmaceutical Group Co., Ltd.; SFDA approval no. H20063851) and 250 ml of sodium chloride injection were injected into the patients by intravenous drip, twice a day. The patients also orally took 0.1 g of aspirin enteric-coated tablets (specification: 100 mg/tablet; manufacturer: Bayer Schering Pharmaceutical Health Co., Ltd.; SFDA approval no. J20130078) once a day and continuously for 12 months. (3) Brain protection: the patients received 30 mg of edaravone injection (specification: 30 mg/vial; manufacturer: Nanjing Simcere Dongyuan Pharmaceutical Co., Ltd.; SFDA approval no. H20031342) and 250 ml of 0.9% sodium chloride injection by intravenous drip, twice a day. (4) Hyperbaric oxygen: hyperbaric oxygen therapy (HBOT) at atmospheric pressure (2.026 × 10^5^ Pa) was performed at 1 hour after thrombolysis, and each time lasted for 1 hour, once a day. (5) Symptomatic treatment: patients with hypertension and diabetes received antihypertensive and hypoglycemic treatment, respectively. In addition, it was necessary to prevent infection and maintain the water-electrolyte balance of patients.

The experimental group was additionally treated with cinepazide maleate. The patients received 240 mg of cinepazide maleate injection (specification: 320 mg/vial; manufacturer: Beijing Sihuan Pharmaceutical Co., Ltd.; SFDA approval no. H20061204) and 250 ml of 0.9% sodium chloride injection by intravenous drip, once a day. The routine treatment was the same with that in the control group. During the treatment, all patients were prohibited from using other cerebral vasodilators, Ca^2+^ antagonists, or nootropic agents. The treatment lasted for 14 days in both groups.

### 2.5. Observation Indexes

#### 2.5.1. Clinical Efficacy

According to the *Clinical Neural Function Deficit Score Criteria for Stroke* [15], the neurological deficit score of patients decreased by more than 90% after treatment, with the disability grade as 0, which was cured. The neurological deficit score decreased by 46%–90%, with the disability grade as levels 1–3, which was markedly effective. The neurological deficit score decreased by 18%–45%, which was improved. The neurological deficit score decreased by less than 17%, which was ineffective. Total effective rate = (improved + markedly effective + cured)/total number × 100%.

#### 2.5.2. Evaluation of Neurological Function

Glasgow Coma Scale (GCS) was used to evaluate the coma degree, including eye opening response (4 points), verbal response (5 points), and motor response of the nonhemiplegia side (6 points), with a total score of 15 points. A score of 8 or less was considered as coma, and a higher score represented a lower level of coma in patients. The National Institutes of Health Stroke Scale (NIHSS) was used to evaluate the neurological deficits, including 11 large dimensions (consciousness, gaze, visual field, facial paralysis, upper limb movement, lower limb movement, ataxia, sensation, language, dysarthria, and neglect), with a total score of 42 points. A higher score represented more serious neurological deficits. Fugl-Meyer motor function measure scale was used to evaluate the comprehensive motor function of patients, with 17 items and a total score of 100 points. The score <50 was considered as severe dyskinesia, 50–84 as obvious dyskinesia, 85–95 as moderate dyskinesia, and 96–99 as mild dyskinesia.

#### 2.5.3. Oxidative Stress Indexes

Fasting venous blood from the elbow was taken in the morning and centrifuged at 4000 r/min for 5 min. After the supernatant was placed in an Eppendorf tube, the total antioxidant capacity (T-Aoc) kits (specification: 50T/48S; brand: Solarbio) were used to detect the T-Aoc levels, superoxide dismutase (SOD) activity kits (specification: 50T/24S; brand: Solarbio) were used to detect the SOD level, glutathione peroxidase (GSH-PX) kits (specification: 50T/343T; manufacturer: Shanghai Caiyou Industrial Co., Ltd.) were used to detect the GSH-PX level, and malondialdehyde (MDA) kits (specification: 100T/96S; brand: Solarbio) were used to detect the MDA level of patients.

Venous blood was collected from patients, and serum was separated. Enzyme-linked immunosorbent assay (ELISA) was used to detect the total antioxidant capacity (T-Aoc), superoxide dismutase (SOD), glutathione peroxidase (GSH-PX), and malondialdehyde (MDA) levels of patients.

#### 2.5.4. Inflammatory Factor Levels

Venous blood was collected from patients to separate serum. Chemiluminescent immunoassay was used to detect the level of high-sensitivity C-reactive protein (hsCRP), and ELISA was used to detect the levels of interleukin-6 (IL-6), interleukin-8 (IL-8), and tumor necrosis factor-*α* (TNF-*α*).

#### 2.5.5. Cerebrovascular Function

A hemodynamic analyzer (model: HM 81-01) was used to detect the vascular function of patients, including the mean cerebral blood flow volume (*Q*_mean_), mean cerebral blood flow velocity (*V*_mean_), peripheral vascular resistance (*R*), and dynamic resistance.

### 2.6. Statistical Treatment

In this study, SPSS 20.0 was selected as data processing software, and GraphPad Prism 7 (GraphPad Software, San Diego, USA) was used to draw pictures of the data. Enumeration data and measurement data were included in the study, tested by *X*^2^, *t*-test, and normality test. The difference was statistically significant when *P* < 0.05.

## 3. Results

### 3.1. Comparison of General Data

There was no significant difference in gender, age, bleeding sites, and other basic information between the two groups (*P* > 0.05), suitable for comparative study, as shown in Table 1.

### 3.2. Comparison of Clinical Efficacy between the Two Groups

The total effective rate in the experimental group was higher than that in the control group (*P* < 0.05), with a statistically significant difference, as shown in Table 2.

### 3.3. Comparison of Neurological Function between the Two Groups

After treatment, the GCS, NIHSS, and Fugl-Meyer scores in both groups were better than those before treatment, and the scores in the experimental group were better than those in the control group, with statistical differences (*P* < 0.05), as shown in Table 3.

### 3.4. Comparison of Oxidative Stress Indexes between the Two Groups

Compared with the control group, T-Aoc, SOD, and GSH-PX in the experimental group were obviously higher, while MDA was lower (*P* < 0.05). All the oxidative stress indexes after treatment were better than those before treatment, with statistical significance (*P* < 0.05), as shown in Table 4.

### 3.5. Comparison of Inflammatory Factor Levels between the Two Groups

After treatment, the hsCRP, IL-6, IL-8, and TNF-*α* levels in both groups were obviously lower than those before treatment, and the levels in the experimental group were lower than those in the control group (*P* < 0.05), with statistical significance, as shown in Table 5.

### 3.6. Comparison of Cerebrovascular Function between the Two Groups

After treatment, the cerebrovascular function in both groups was obviously improved, and the function in the experimental group was obviously better than that in the control group (*P* < 0.05), as shown in Table 6.

## 4. Discussion

Hypertensive cerebral hemorrhage (HICH) is a common high-risk disease in clinics, and most patients in clinics mainly receive medical treatment. If patients with surgical indications have more serious condition or their secondary cause is found, surgical treatment will be adopted to mainly reduce intracranial pressure, remove hematoma, and save the life of patients. In addition, patients need to control blood pressure to reach the standard and be stable for life [16]. The prognosis of the disease is often related to the amount of bleeding, bleeding sites, and complications. Patients are considered to have good prognosis if they experience a small amount of blood loss with no bad complications during treatment, and their bleeding sites do not affect the neurological function. Patients have poor prognosis if they suffer from complications such as pulmonary infection and gastrointestinal bleeding [17–20]. Clinical statistics suggest that severe intracerebral hemorrhage can account for about half of intracerebral hemorrhage cases. Failure to take timely and effective measures will directly affect the recovery of patients after intervention, leading to sequelae or even death. In recent years, the medical research about cinepazide maleate mostly focuses on its effect on HICH and lacks studies on severe cerebral hemorrhage. Therefore, this paper retrospectively analyzed the clinical data of 116 ICU patients with severe cerebral hemorrhage treated in our hospital, observed their serum inflammatory factor levels, and explored the clinical effect of cinepazide maleate on the patients, neurological function, inflammatory response, and oxidative stress injury, aiming to provide a reference for the optimization of clinical therapeutic schedules for ICU patients with severe cerebral hemorrhage.

Cinepazide maleate injection is a Ca^2+^ antagonist that can prevent Ca^2+^ from penetrating into vascular smooth muscle cells across the membrane and relax the vascular smooth muscle, thereby expanding cerebral, peripheral, and coronary vessels to relieve vasospasm, reduce vascular resistance, and increase blood flow. In addition, cinepazide maleate can enhance the role of cyclic adenosine monophosphate and adenosine, reduce oxygen consumption, and increase the content of cyclic adenosine monophosphate by inhibiting cAMP phosphodiesterase. In addition, it can improve the deformability and flexibility of red blood cells to enhance their ability to pass through small blood vessels, thereby reducing blood viscosity and improving microcirculation [21–24]. This study showed that the total effective rate in the experimental group was higher than that in the control group, indicating that cinepazide maleate can improve the postoperative therapeutic effect of patients with cerebral hemorrhage compared with routine treatment. After treatment, the GCS, NIHSS, and Fugl-Meyer scores in both groups were better than those before treatment, and the scores in the experimental group were better than those in the control group (*P* < 0.05). GCS was mainly used to evaluate the coma degree of patients with cerebral hemorrhage, NIHSS was to evaluate the neurological deficits, and Fugl-Meyer reflected the comprehensive motor function. It can be seen that cinepazide maleate can effectively enhance the postoperative neurological function of patients, improve brain metabolism, and promote the recovery of brain function. The oxidative stress indexes such as T-Aoc, SOD, and GSH-PX in the experimental group were higher than those in the control group, while MDA in the experimental group was lower than that in the control group. The hsCRP, IL-6, IL-8, and TNF-*α* levels in the experimental group were lower than those in the control group. Compared with the control group, the cerebrovascular function in the experimental group was significantly improved. Oxidative stress response and inflammatory response are closely related to the pathological changes of nerve injury and edema in patients with cerebral hemorrhage. After cerebral hemorrhage, hematoma occurs rapidly in the lesion area, resulting in the death of a large number of brain nerve cells around the lesions. At the same time, the blood supply area of the bleeding vessel forms reperfusion injury which produces lots of inflammatory factors and then leads to systemic inflammatory response. The further development of inflammation will bring about microglia activation, infiltration of inflammatory cells around the lesions, and release of proinflammatory mediators, eventually resulting in cell death and brain injury. If the inflammatory response is not timely controlled, it will also aggravate the risk of secondary injury after cerebral hemorrhage. When cerebral hemorrhage occurs, the brain tissue will also suffer from oxidative damage, which is a potential damage state in which the oxides and antioxidants in the body lose their dynamic balance. Under the common effect of inflammatory factors, lots of oxygen free radicals are generated in the lesion area, aggravating the damage of surrounding nerve cells. In addition, oxygen free radicals can also form the blood-brain barrier, causing systemic oxidative stress injury. Therefore, it is of great significance to improve the inflammatory factor levels and oxidative stress response for the postoperative treatment of patients. In summary, the implementation of cinepazide maleate-combined routine treatment after surgery has a positive effect on patients with severe cerebral hemorrhage, which can improve the cerebral blood flow, promote microcirculation, and have good anti-inflammatory effect, thereby reducing cerebral damage. Jia et al. [25] believed that cinepazide maleate had the effect of reducing serum inflammatory factor levels and blood viscosity and had a good clinical therapeutic effect on cerebral hemorrhage, which is consistent with the results of this study. The study has some shortcomings. For example, it is a single-center study with a small sample size, and the clinical efficacy of cinepazide maleate needs to be further verified by multicenter studies with an expanded sample size. In addition, this study lacks the observation and analysis of the long-term efficacy of patients.

In conclusion, cinepazide maleate can effectively reduce the serum inflammatory factor levels of ICU patients with severe cerebral hemorrhage after surgery, alleviate the oxidative stress response in the body, and improve the cerebrovascular function and cerebral nerve function, which is worthy of clinical promotion.

## Figures and Tables

**Table 1:** Comparison of basic data between the two groups.

Items	Control group (*n* = 58)	Experimental group (*n* = 58)	*t*/*X*^2^	*P*
Age (years old)	63.5 ± 7.32	62.8 ± 7.09	0.523	0.602
BMI (kg/m^2^)	25.57 ± 5.18	25.51 ± 5.06	0.063	0.950
Amount of bleeding (ml)	42.85 ± 4.57	43.04 ± 4.77	0.219	0.827
Systolic pressure (mmHg)	121.36 ± 9.73	120.68 ± 9.67	0.378	0.707
Diastolic pressure (mmHg)	95.32 ± 6.24	94.81 ± 6.33	0.437	0.663
Gender	—	—	0.153	0.696
Male	37 (63.79%)	39 (67.24%)		
Female	21 (36.21%)	19 (32.76%)		

Bleeding sites				
Basal ganglia	43 (74.14%)	45 (77.59%)	0.188	0.664
Thalamus	11 (18.97%)	10 (17.24%)	0.058	0.809
Others	4 (6.90%)	3 (5.17%)	0.152	0.691

Concomitant diseases				
Hypertension	17 (29.31%)	20 (34.48%)	0.357	0.550
Diabetes mellitus	11 (18.97%)	10 (17.24%)	0.058	0.809

**Table 2:** Comparison of clinical efficacy between the two groups (*n* (%)).

Group	Ineffective	Improved	Markedly effective	Cured	Total effective rate
Control group (*n* = 58)	15 (25.86)	16 (27.59)	14 (24.14)	13 (22.41)	43 (74.14)
Experimental group (*n* = 58)	6 (10.34)	11 (18.97)	20 (34.48)	21 (36.21)	52 (89.66)
*X* ^2^	—	—	—	—	4.710
*P*	—	—	—	—	0.030

**Table 3:** Comparison of neurological function between the two groups (*n* = 58, $\bar{x}$ ± *s*).

Group	GCS score		NIHSS score		Fugl-Meyer score	
	Before treatment	After treatment	Before treatment	After treatment	Before treatment	After treatment
Control group	6.25 ± 0.58	10.98 ± 1.33	16.97 ± 1.74	10.41 ± 1.09	43.88 ± 4.25	60.64 ± 6.71
Experimental group	6.18 ± 0.61	14.71 ± 1.37	17.32 ± 1.78	7.46 ± 0.73	44.15 ± 4.31	71.57 ± 7.47
*t*	0.633	14.877	0.071	17.126	0.340	8.290
*P*	0.528	<0.05	0.287	<0.05	0.735	<0.05

**Table 4:** Comparison of oxidative stress indexes between the two groups ($\bar{x}$ ± *s*).

Indexes		Control group (*n* = 58)	Experimental group (*n* = 58)	*t*	*P*
T-Aoc (U/L)	Before treatment	0.94 ± 0.08	0.96 ± 0.08	1.346	0.181
	After treatment	1.78 ± 0.22	3.15 ± 0.36	24.730	<0.05

SOD (U/L)	Before treatment	14.05 ± 1.19	13.68 ± 1.17	1.689	0.094
	After treatment	55.71 ± 5.72	86.19 ± 8.85	22.029	<0.05

GSH-PX (U/L)	Before treatment	89.65 ± 9.43	90.12 ± 9.52	0.267	0.790
	After treatment	150.41 ± 15.07	197.36 ± 19.86	14.342	<0.05

MDA (nmol/L)	Before treatment	3.74 ± 0.38	3.69 ± 0.35	0.737	0.463
	After treatment	2.14 ± 0.25	1.61 ± 0.18	13.103	<0.05

**Table 5:** Comparison of inflammatory factor levels between the two groups ($\bar{x}$ ± *s*).

Indexes		Control group (*n* = 58)	Experimental group (*n* = 58)	*t*	*P*
hsCRP (mg/L)	Before treatment	3.14 ± 0.53	3.26 ± 0.58	1.163	0.247
	After treatment	1.59 ± 0.20	1.04 ± 0.15	16.755	<0.05

IL-6 (ng/L)	Before treatment	124.09 ± 12.38	123.85 ± 12.51	0.104	0.918
	After treatment	89.42 ± 8.71	45.31 ± 8.03	29.315	<0.05

IL-8 (ng/L)	Before treatment	5.61 ± 0.55	5.68 ± 0.57	0.673	0.502
	After treatment	1.98 ± 0.35	1.35 ± 0.23	11.456	<0.05

TNF-*α* (*µ*g/L)	Before treatment	2.18 ± 0.43	2.17 ± 0.40	0.130	0.897
	After treatment	1.29 ± 0.31	0.92 ± 0.22	7.413	<0.05

**Table 6:** Comparison of cerebrovascular function between the two groups ($\bar{x}$ ± *s*).

Indexes		Control group (*n* = 58)	Experimental group (*n* = 58)	*t*	*P*
*Q*_mean_ (ml/s)	Before treatment	8.4 ± 0.6	8.5 ± 0.7	0.826	0.411
	After treatment	10.3 ± 7.1	14.7 ± 7.8	3.177	0.0019

*V*_mean_ (cm/s)	Before treatment	12.2 ± 1.2	12.3 ± 1.3	0.430	0.668
	After treatment	15.7 ± 1.5	18.2 ± 1.9	7.865	<0.05

*R* (kPa·s/m)	Before treatment	1963.1 ± 164.2	1968.4 ± 165.1	0.173	0.823
	After treatment	991.8 ± 90.2	874.1 ± 88.3	7.101	<0.05

Dynamic resistance (kPa·s/m)	Before treatment	472.3 ± 47.1	469.7 ± 45.6	0.302	0.763
	After treatment	385.9 ± 40.1	311.5 ± 32.2	11.018	<0.05

## Data Availability

The data used to support the findings of this study are available from the corresponding author upon reasonable request.
